# Region-Based Segmentation and Classification for Ovarian Cancer Detection Using Convolution Neural Network

**DOI:** 10.1155/2022/5968939

**Published:** 2022-11-19

**Authors:** L. K. Hema, R. Manikandan, Majid Alhomrani, N. Pradeep, Abdulhakeem S. Alamri, Shakti Sharma, Musah Alhassan

**Affiliations:** ^1^Department of Electronics and Communication Engineering, Aarupadai Veedu Institute of Technology, Vinayaka Mission& Research Foundation, Salem, Tamil Nadu, India; ^2^School of Computing, SASTRA Deemed University, Thanjavur, India; ^3^Department of Clinical Laboratories Sciences, The Faculty of Applied Medical Sciences, Taif University, Taif, Saudi Arabia, and Centre of Biomedical Sciences Research (CBSR) Deanship of Scientific Research, Taif University, Taif, Saudi Arabia; ^4^Department of Computer Science and Engineering, Bapuji Institute of Technology, Davangere, Karnataka, India; ^5^School of Computer Science Engineering & Technology, Bennett University, Greater Noida, India; ^6^University of Development Studies, Electrical Engineering Department, School of Engineering, Nyankpala Campus, Nyankpala, Ghana

## Abstract

Ovarian cancer is a serious sickness for elderly women. According to data, it is the seventh leading cause of death in women as well as the fifth most frequent disease worldwide. Many researchers classified ovarian cancer using Artificial Neural Networks (ANNs). Doctors consider classification accuracy to be an important aspect of making decisions. Doctors consider improved classification accuracy for providing proper treatment. Early and precise diagnosis lowers mortality rates and saves lives. On basis of ROI (region of interest) segmentation, this research presents a novel annotated ovarian image classification utilizing FaRe-ConvNN (rapid region-based Convolutional neural network). The input photos were divided into three categories: epithelial, germ, and stroma cells. This image is segmented as well as preprocessed. After that, FaRe-ConvNN is used to perform the annotation procedure. For region-based classification, the method compares manually annotated features as well as trained feature in FaRe-ConvNN. This will aid in the analysis of higher accuracy in disease identification, as human annotation has lesser accuracy in previous studies; therefore, this effort will empirically prove that ML classification will provide higher accuracy. Classification is done using a combination of SVC and Gaussian NB classifiers after the region-based training in FaRe-ConvNN. The ensemble technique was employed in feature classification due to better data indexing. To diagnose ovarian cancer, the simulation provides an accurate portion of the input image. FaRe-ConvNN has a precision value of more than 95%, SVC has a precision value of 95.96%, and Gaussian NB has a precision value of 97.7%, with FR-CNN enhancing precision in Gaussian NB. For recall/sensitivity, SVC is 94.31 percent and Gaussian NB is 97.7 percent, while for specificity, SVC is 97.39 percent and Gaussian NB is 98.69 percent using FaRe-ConvNN.

## 1. Introduction

One of the most common types of cancer in women is Ovarian Cancer (OC). In year 2018, 295,414 women were diagnosed with ovarian cancer, which resulted in 184,799 deaths around the world. Since early-stage tumors are often asymptomatic, most women with ovarian cancer have advanced disease at the time of diagnosis, resulting in a lower long-term survival [1]. Although ovarian tumors are chemosensitive as well as exhibit initial success against platinum/taxane treatment, the 5-year recurrence rates in patients with advanced illness are 60 percent to 80 percent [2].

It is characterized by early-stage symptoms that are modest and a low survival rate. The most common as well as dangerous gynecologic cancer is OC. Serous, mucinous, Endometroid, and clear cell ovarian cancer are four subtypes of primary epithelial ovarian carcinoma [3]. According to earlier research, one out of every 54 women can acquire OC.5-year survival rate for a patient diagnosed with OC is roughly 48.6%[4]. The low survival rate is largely attributable to cancer discovery at an advanced stage, with 72 percent of patients diagnosed at stage III or IV. As a result, early detection is critical. Attempts to detect OC in the preclinical stage have been made in the past, employing both medical imaging and blood markers. Although these biomarkers show promise, they have a number of drawbacks, including missing classification, sluggishness, and longer working hours [5].

Although the Serum Carbohydrate Antigen (CA125) is commonly utilized, its accuracy rate is low due to its high sensitivity. Ultrasound imaging, MRI, and CT scan are some of the imaging modalities that are used to locate and characterize tumors. Early detection of any medical condition, particularly cancer, is critical for improving survival rates. Medical imaging is one of the most successful ways for early-stage diagnosis, prediction of brain imaging modalities, monitoring cancer stages, and follow-up procedures after cancer therapy, according to studies. Manually interpreting the data from these medical photographs is time-consuming and prone to human error [6]. The normal ovary and origin of three types of ovarian cancer have been shown in Figure 1. There are three main types of ovarian tumors.

### 1.1. Epithelial Tumors

This type of tumors is derived from the cells on the surface of the ovary. This is the most common form of ovarian cancer and occurs primarily in adults.

### 1.2. Germ Cell Tumors

This type of tumors is derived from the egg producing cells within the body of the ovary. This occurs primarily in children and teens and is rare by comparison to epithelial ovarian tumors.

### 1.3. Stromal tumors

These tumors are rare in comparison to epithelial tumors and this class of tumors often produces steroid hormones.

In addition, computer-aided diagnosis (CAD) methods are frequently employed to assist physicians and pathologists in better analyzing the outcomes of medical images. ML methods are employed in a CAD-based medical imaging strategy for cancer detection [7]. Feature extraction is a crucial stage in the machine learning approach [8]. In the literature, many feature extraction approaches have been examined and analyzed in the context of various MRI, CT, and ultrasound images. Previous work has focused on generating worthy feature descriptors and ML methods for context learning from various types of medical images. These methods have some drawbacks that limit the use of CAD-based medical diagnostic procedures. In this study, we focus on representation learning rather than a learning-based strategy to solve the shortcomings of CAD-based systems. Deep Learning learns from image data using hierarchical feature representation, a form of representation learning technique [9]. The image data itself is used to produce high-level feature representation. The deep learning approach has gained huge profits and success in different applications like image recognition, objection detection, speech processing, and many others [10] with the addition and support of considerable parallel architecture and GPU. Physicians classify patients' symptoms into one of several illness classes based on their understanding. Learning categorization model is a learning challenge in this study for ovarian problems. A broad classification approach was discovered through data analysis. Training data containing cases such as objects or instances is characterized using attribute vectors (features or variables). It could be either quantitative or qualitative in nature. In supervised learning, mutually exclusive cases, as well as class data, are employed for learning, when all cases have the same attribute vector from the same class.

## 2. Literature Survey

Recent research [9] has demonstrated that combining genetic data with pathology images to diagnose tumors is very effective. For predicting breast cancer outcome, researchers [10] combined pathology images and genetic data. To connect the heterogeneous data of two modalities, a multiple kernel learning method was used. Method had an accuracy of 0.8022 and a precision of 0.7273. M2DP, a multi-modal task feature selection technique for cancer diagnosis, was introduced in [11]. Method was tested utilizing a breast cancer benchmark and a lung cancer benchmark, with an accuracy of 72.53 percent and 70.08 percent. In [12], the author proposed a various kernel strategies for forecasting lung carcinomas by combining genomic data with pathological aspects of images, with an accuracy of 0.8022 [13]. Using a DL model, the machine fully extracted deep features from the gene as well as image modalities, and then combined the disparate features utilizing weighted linear aggregation. The accuracy of prediction was 88.07 percent. Recent developments in CNN and other DL methods have profound implications in medical diagnostics. For histopathologic analysis of prostate cancer, the author [14] used a deep residual CNN. The model correctly classified the image patches into benign and malignant at a coarse level of 91.5 percent of the time. Using residual networks, study [15] presented a method for automatically classifying brain cancers (ResNet50 architecture). On a patient-by-patient basis, the model accuracy was 0.97. For classifying dermoscopy images, author [16] utilized deep GoogleNet Inception. Precision was 0.677 [17]. DenseNet-161 and ResNet-50 were used in this study. The *F*-score of the DenseNet-161 model was 92.38 percent, while the accuracy was 91.57 percent. However, many jobs in the realm of medical applications are reliant on long-range interdependence [18]. RNN methods are the most popular approaches for learning longitudinal data in depth. LSTM [19] is an RNN version that captures both LSTM dependencies within sequential input. The F-score for the method was 0.8905 [20].  Table 1 depicts the comparative analysis of proposed and existing techniques.

## 3. Research Methodology

This section discusses the proposed technique in ovarian cancer detection based on segmentation and classification using deep learning architectures. Overfitting and other errors might occur if the training sample is too small. To enhance classification accuracy, we increased the sample size in our study by manipulating images [22]. Image enhancement and rotation are examples of image manipulation. To improve sample sizes, we rotated original input images from 0° to 270° in 90° steps around their center point. Our two groups of data produced two separate recognition models [23]: one used the original image dataset as training data without image segmentation and other utilized the image dataset as training data, with a sample size 11 times larger than the original image dataset.  Figure 2 depicts the architecture of this study process [24].

The input image was divided into three categories: epithelial, germ, and stroma cells. The image is first preprocessed for noise reduction as well as filtering. This image was manually tagged as well as trained utilizing the standard training model [25]. This study used a NN known as the FaRe-ConvNN to compensate for hand annotation. Using FaRe-ConvNN, an object is detected using a trained image and a manually segmented image. Since the convolution is used to detect edges, both features are annotated based on region. Image segmentation has annotated contextual features. The accuracy of disease detection utilizing computer-assisted diagnosis is higher than that of manual detection. Gaussian NB and SVC are utilized for classification when FaRe-ConvNN is applied [26].

Through various processing techniques or combinations of multiple processing, such as random rotation, shifts, shear, flips, etc., image augmentation artificially generates training images. The validation error must drop along with the training error in order to create useful Deep Learning models. This can be done very well with data augmentation. The distance between the training and validation sets, as well as any upcoming testing sets, will be minimized because the augmented image will represent a wider range of potential image locations. The suggested method seeks to enhance segmentation outcomes by creating a new MRI image dataset from an existing MRI image dataset. In this work, the segmentation of the ovarian imaging collection is specifically discussed. It is stated that the segmentation task entails locating the pixels that belong to the ovarian cancer image and separating the nuclei from the surrounding tissue. We can totally rearrange the pixels in an image enhancement process that involves flipping an image horizontally or vertically while maintaining the features. Images may be at a range of angles, though they are unlikely to be upside down. Each image may be rotated by a different amount. The majority of the image's pixel values have changed from the original image's values.

Incorrect pixel values that are randomly distributed throughout the image can also be used to add noise to the image. Each image in the training set can be enhanced using standard augmentation methods like flips and rotations without requiring manual image processing. Batches of photos are pulled from the directory by “ImageDataGenerator,” which then applies transformations like “vertical flip,” “horizontal flip,” or “rotation range.”

The enhanced images first go through pre-processing to improve them before computation. The pre-processing step primarily results in the collection of images under various methods of image examination. It changes the applied image into a new one that is essentially identical to the applied image, with a few minor differences. Resizing, masking, segmentation, normalization, noise removal, and other pre-processing procedures are some of them. By downsizing the photos and filtering the noises that are present in the image, this study preprocesses the applied product images. Each image is changed to its default size of 300 × 300 pixels before being resized. Resized photographs are sent to the filtering process so that the product images can produce better results.

### 3.1. Cancer Detection Using FaRe-ConvNN

#### 3.1.1. Convolution Layer

A set of filters make up the convolutional layer. The learnable parameters of layer are the values of these filters. When it comes to CNNs, the goal behind convolution is to extract features from an image while keeping the spatial relationship between pixels as well as learnt features inside the image by using small, equal-sized tiles. For an *MN* 3 input image with *K* filters of size I *J* in the first convolutional layer, where *I* <<< *N* and 3 indicate the color channels. Every element from input image as well as filter matrix undergoes a mathematical process, which results in the learned features [4]. This is what it means:

(1) $$\begin{array}{c} x_{i,j}^{l}=\sum_{a}\sum_{b}w_{a,b}^{\left(l-1,f\right)}y_{i+a,j+b}^{\left(l-1\right)}+\text{bias }f, \end{array}$$

where *y*_*i*,*j*_^*l*^ is output of layer *l*, *w*_*a*,*b*_^(*l* − 1, *f*)^ is weight of filter *f* which is used at layer l-1. To put it another way, the filter slides through all of the image's elements and multiplies each one, resulting in a single matrix called a feature map. Size of the feature map matrix is determined by the depth and stride.

Additionally, an activation function known as ReLU is commonly utilized to introduce non-linearity to CNNs, allowing them to learn nonlinear models. This rectifier approach is most commonly utilized since ReLU considerably enhances CNN object identification performance [27].

#### 3.1.2. Pooling Layer

Pooling is one of ConvNet's unique concepts, as previously noted. Pooling step's goal is to lower the dimensionality of every feature map by removing noisy, unnecessary convolutions and computation networks while keeping the majority of the critical data. There are several types, including Max, Sum, and Average, but max-pooling is the most popular and recommended [28]. In max-pooling, a spatial neighborhood is constructed, and the max unit is obtained from the feature map depending on the filter dimension, which are 2×2 windows, for example.  Figure 3 displays max-pooling with a 2×2 window as well as a stride of 2, which reduces the dimensionality of the Feature Map by picking the maximum of each region.

#### 3.1.3. Fully Connected Layer

It comes directly before the output layer in a ConvNet and functions like a standard NN at end of convolutional as well as pooling layers. Each neuron on a fully connected layer is coupled to each neuron on the layer before the FC layer. The FC Layer's goal is to utilize the preceding layer's output features to classify images using the training dataset. In essence, a CNN's fully connected layers act as a classifier, with convolutional layer outputs serving as classifier's input [29].

Figure 4 shows the unified structure of FaRe-ConvNN and RPN. Modern object detectors have anchor boxes as a standard feature. A rectangular box is acquired for every object in an image during object detection, resulting in many boxes of varied shapes as well as sizes in every image.

The images are first separated into grids. The reason for this is that medical photographs are typically quite large. You also want to make sure that each grid has labeling (done by specialists). CNN [30] is trained on each grid. Each grid is provided with a mask that states “cancerous” or “non-cancerous” when it is transmitted. Then, as you glide through each grid, train the NN to recognize each grid's mask.

#### 3.1.4. Region Proposal Network

Feature map is RPN's input, while the output is a series of rectangular object proposals, each with an objectless score [31]. The selective search takes 2 seconds per image to propose a region, whereas RPN takes only 10 ms. Anchor boxes with three aspect ratios and three scales are used by FaRe-ConvNN. As a result, there are 9 anchor boxes for every pixel in the feature map. A simple convolution layer with a kernel size of 3*∗*3 is followed by two FC layers in the architecture. 1*∗*1 convolutional layers are used to create this fully connected layer. The classification layer's output size should be 2*∗*9, whereas the regression layer's output size should be 4*∗*9. For each pixel in the feature map, the total number of predictions [32] will now be (4 + 2)*∗*9*∗*(*H∗W*).

#### 3.1.5. Loss Function

Loss function utilized in FR-CNN is represented by the following:

(2) $$\begin{array}{c} L\left(\left\{p_{i}\right\},\left\{t_{i}\right\}\right)=\frac{1}{N_{\text{cls}}}\sum_{j}^{m}ZL_{\text{cls}}\left(p_{i},p_{i}^{*}\right)+\lambda \frac{1}{L_{\text{reg}}}\sum_{i}^{n}Yp_{i}^{*}L_{\text{cls}}\left(p_{i},p_{i}^{*}\right). \end{array}$$

As previously stated, regression offset is determined using the closest anchor box. Anchor boxes are now acting as region proposals, which is related to the region proposal technique. At training time, all anchor boxes do not contribute to loss. Positive labels are given to anchors with the biggest IOU with ground truth as well as IOU overlap greater than 0.7. The training purpose is not served by anchors that are neither positive nor negative. Anchors that cross borders are also ignored [33].

Consider data {*y*_*j*_} with labels {*z*_*j*_} such that ×={(*y*_*j*_, *x*_*j*_)*|y*_*j*_ ∈ *R*^*m*^, *z*_*j*_ ∈ *R*^*n*^, *j*=1,…*M*} a FaRe-ConvNN finds function *f*_DNN_ : *R*^*m*^⟶*R*^*n*^ to weave via data such that *f*_DNN_(*y*_*j*_)≅*z*_*j*_ as much as possible through the utility of 3 various parts: An activation function *ρ* : *R*^*m*_*i*−1_^⟶*R*^*m*˙_*i*_^*x*^(*i* − 1)^ ∈ *R*^*m*_*i*−1_^ would satisfy by the following:

(3) $$\begin{array}{c} x^{\left(i\right)}=\rho \left(\Theta^{\left(i-1\right)}\cdot x^{\left(i-1\right)}+a^{\left(i-1\right)}\right). \end{array}$$

Objective function is Min(*F*) from (4) where

(4) $$\begin{array}{c} F=\text{Min}\left[\text{Min}\left(\sum_{x=1}^{x}\text{Min}\left(f_{1}\right)\right)-\text{Min}\left(f_{2}\right)+\text{Min}\left(f_{3}\right)\right], \end{array}$$

where

(5) $$\begin{array}{c} f_{1}=\text{Min}\left(\sum_{i=1}^{l}\sum_{y=1}^{Y}\sum_{z=1}^{z}\left(t_{ixyz}\right)\left(l_{ixyx}\right)\right)f_{2}=\text{Max}\left(\frac{I*X}{\sum_{i=1}^{l}\sum_{x=1}^{X}\sum_{y=1}^{Y}\sum_{z=1}^{Z}\left(t_{ixyz}\right)\left(l_{ixyx}\right)}\right)\\ f_{3}=\text{min}\left(\sum_{i=1}^{1}\sum_{y=1}^{Y}\sum_{z=1}^{z}\left(l_{ixyz}\right)\left(t_{ixyz}\right)-\sum_{i=1}^{1}\sum_{y=1}^{Y}\sum_{z=1}^{z}\left(l_{i\left(x+1\right)yz}\right)\left(t_{i\left(x+1\right)yz}\right)\right)\approx 0\forall M_{x},x\\ =1,2,\left(X-1\right)=1,L,,\left(x-1\right). \end{array}$$

Decision variables and constraints have been given by following:

(6) $$\begin{array}{c} \sum_{y=1}^{Y}\sum_{x=1}^{X}\sum_{z=1}^{z}\left(l_{ixyz}\right)=\sum_{y=1}^{Y}\sum_{x=1}^{X}\left(M_{ixy}\right)\left(To_{ixy}\right)\forall O_{y}\text{ of }J_{i}\text{ and }i,i=1,2,I\&y\\ =1,2,Y\sum_{x=1}^{X}\sum_{z=1}^{z}l_{ixyz}=\sum_{x=1}^{x}\left(M_{ixy}\right)\left(To_{ixy}\right)\forall O_{y}\&J_{i},i=1,2,I\&y=1,2,Y\sum_{x=1}^{x}\left(M_{ixy}\right)\\ =1\forall O_{y}\text{ of }J_{i},\text{and}i,i=1,2,I\&y=1,2,Y. \end{array}$$

Consider an affine approximation to *f*(*X*) = ‖*Y* − *H*_*c*_*XH*_*r*_^*⊤*^‖_*F*_^2^ in (2) at *X*^*l*^ and the following update rule:

(7) $$\begin{array}{c} X^{l+1}=\text{arg}\underset{X}{\text{min}}f\left(X^{l}\right)+Tr{\left(X-X^{l}\right)}^{⊤}\nabla f\left(X^{l}\right)+\frac{1}{2\eta }{\left\|X-X^{l}\right\|}_{F}^{2}+\lambda G\left(X\right), \end{array}$$

where ‖*X* − *X*^*l*^‖_*F*_^2^ serves as proximal term is expressed as follows:

(8) $$\begin{array}{c} X^{l+1}=P_{\nu }\left(X^{l}-\eta \nabla f\left(X^{l}\right)\right), \end{array}$$

where *P*_*ν*_ is the proximal operator corresponding to *G* and *ν* = *λη*. From (9) and (10), proximity operator is defined.

(9) $$\begin{array}{c} G\left(X\right)={\left\|X\right\|}_{1}≜\sum_{i=1}^{M}\sum_{j=1}^{N}\left|X_{i,j}\right|. \end{array}$$

(10) $$\begin{array}{c} P_{\nu }\left(X_{ij}\right)=\text{sgn}\left(X_{ij}\right)m\left\{\left|X_{ij}\right|-\nu ,0\right\}, \end{array}$$

where sgn(·) denotes signum function. The update that results is identical to usual iterative ISTA. Utilizing 11 gradient expression,

(11) $$\begin{array}{c} \nabla f\left(X\right)=H_{c}^{⊤}\left(H_{c}XH_{r}-Y\right)H_{r}^{⊤}. \end{array}$$

Equation (12)is expressed in following form:

(12) $$\begin{array}{c} X^{l+1}=P_{\nu }\left(X^{l}-\eta H_{c}^{⊤}H_{c}X^{l}H_{r}H_{r}^{⊤}+C\right). \end{array}$$

The activation function *ψ* is defined as a linear combination of K DoG, and linear function is defined as the following equations:

(13) $$\begin{array}{c} \psi \left(u\right)=\sum_{k=1}^{K}c_{k}\phi_{k}\left(u\right),u\in R, \end{array}$$

where

(14) $$\begin{array}{c} \phi_{k}\left(u\right)=u\text{exp}\left(-\frac{\left(k-1\right)u^{2}}{2\tau^{2}}\right). \end{array}$$

Training dataset *D* contains *N* examples {(*Y*_*q*_, *X*_*q*_)}_*q*=1_^*N*^, where *Y*_*q*_=*H*_*c*_*X*_*q*_*H*_*r*_^*⊤*^+*ξ*_*q*^*∗*^_ Random noise vectors *ξ*_*q*_ are considered to be equally distributed as well as independent. Let *c*^*l*^ ∈ *R*^*K*^, *l*=1 be coefficients of LET activation in layer [34]. By reducing squared estimation error over all training examples, the optimal set of activation specifications c^*∗*^ is obtained as follows:

(15) $$\begin{array}{c} J\left(c\right)=\frac{1}{2}\sum_{q=1}^{N}{\left\|X_{q}^{L}\left(Y_{q},c\right)-X_{q}\right\|}_{2}^{2}. \end{array}$$

Gradient of *J* (*c*) with respect to *c* is required for optimization. Unless a very tiny step size is specified, optimization of *J* (*c*) utilizing vanilla GD tends to diverge. We get around this problem by pointing out that the Hessian does not have to be computed directly. To train the network's parameters, all that is required is the Hessian-vector product. Search direction *δ*_*c*_^*∗*^ is determined in *I*th iterate ci of HFO by minimizing a second-order Taylor-series approximation *J*˜(*c*) to actual cost *J* (*c*) by the following:

(16) $$\begin{array}{c} J\tilde{\left(c_{i}+\delta_{c}\right)}=J\left(c_{i}\right)+\delta_{c}^{⊤}g_{i}+\frac{1}{2}\delta_{c}^{⊤}H_{i}\delta_{c}, \end{array}$$

where *g*_*i*_=∇*J*(*c*)*|*_*c*=*c*_*i*__, *H*_*i*_=∇^2^*J*(*c*)*|*_*c*=*c*_*i*__, and *δ*_*c*_ is search direction to be selected optimally at each iteration by reducing a normalized quadratic approximation by (17):

(17) $$\begin{array}{c} \delta_{c}^{*}={\text{argmin}}_{\delta_{c}}J\tilde{\left(c_{i}+\delta_{c}\right)}+\gamma {\left\|\delta_{c}\right\|}_{2}^{2}.\\ X_{t+1}=X_{t}+\text{Lévy}\left(d\right)\times X_{t}\\ \text{Lévy}\left(x\right)=0.01\times \frac{r_{1}\times \sigma }{{\left|r_{2}\right|}^{1/\beta }}\\ \sigma ={\left(\frac{\Gamma \left(1+\beta \right)\times \text{sin}\left(\pi \beta /2\right)}{\Gamma \left(1+\beta /2\right)\times \beta \times 2^{\left(\beta -1/2\right)}}\right)}^{1/\beta }. \end{array}$$

The dimension of the position vectors is *d*. In the range [0, 1], *R*1, *r*2 are two random values, *β* is a constant, and Γ(x) = (x − 1)! Equation (18) is used to determine the fitness function here:

(18) $$\begin{array}{c} {\text{fit}}_{i}=\frac{1}{1+f_{i}}\\ f_{i}=\frac{1}{n_{j}}\sum_{i=1}^{nj}d\left(X_{j},C_{i}\right). \end{array}$$

The level set function *ϕ* is a surface that is positive inside region *Ω*, negative outside the region *Ω*, defined over image space. The level set equation in its most general form is as follows:

(19) $$\begin{array}{c} \frac{\partial \varphi }{\partial t}=-F.\left|\nabla \varphi \right|,\varphi \left(x,y,t=0\right)\\ =\pm \text{d}F=-\alpha k\cdot g-\beta \cdot g-\lambda \nabla g\cdot \frac{\nabla \varphi }{{\left|\nabla \varphi \right|}^{\prime }}g=\frac{1}{1+{\left|\left(\nabla G_{\sigma }\right)⊗I\left(X\right)\right|}^{\beta }}G_{\sigma }\left(\varepsilon \right)\\ =\frac{1}{\sqrt[{n}]{\pi }}e^{-\left(\varepsilon /\sigma \right)2}\frac{\partial \varphi \left(x,y,t\right)}{\partial t}\\ =\alpha k\cdot g\left(x,y\right)\cdot \left|\nabla \varphi \right|+\beta \cdot g\left(x\cdot y\right)\cdot \left|\nabla \varphi \right|+\lambda \cdot \nabla g\cdot \nabla \varphi \\ \left\{\varphi \left(X,t\right)>0,\text{if }X\in \Omega \varphi \left(X,t\right)=0,\text{ if }X\in \Gamma ,\varphi \left(X,t\right)<0,\text{otherwise}\right.. \end{array}$$

#### 3.1.6. Training

A CNN should be trained on a large database of images in order to attain low error rates. Backpropagation is utilized to train CNN by computing the gradient required for updating the network's weights. Depending on which layer is being taught, there are number of different steps to train the CNN [35].

The backpropagation mechanism is used in the FC layer. The squared error loss function, as shown in (1), must first be used to estimate the error or cost function indicated E(yL) at the output layer as follows:

(20) $$\begin{array}{c} E^{N}=\frac{1}{2}\sum_{n=1}^{N}\sum_{k=1}^{c}{\left({\text{target}}_{k}^{n}-y_{k}^{n}\right)}^{2}, \end{array}$$

target_*k*_^*n*^ is the *n*th training example target of class *k*, while *y*_*k*_^*n*^ is the actual output from last layer.

Derivative of error function is partial derivative from output layer [25], as shown in the following:

(21) $$\begin{array}{c} \frac{\partial^{1}}{\partial y_{i}^{L}}=\frac{d^{1}}{dy_{i}^{L}}E\left(y^{L}\right). \end{array}$$

For every input to current neuron, (*∂E*/*∂x*_*j*_^1^) usually known as delta must be determined.

(22) $$\begin{array}{c} \frac{\partial E}{\partial x_{j}^{1}}=\sigma^{\prime }\left(x_{j}^{1}\right)\frac{\partial E}{\partial y_{i}^{1}}. \end{array}$$

*σ*(*x*_*j*_^1^) relates ReLU function *σ* is used to *x*_*j*_^1^ which is input to the current neuron. After you've completed this for all neurons, you'll need to calculate the errors from the previous layer.

(23) $$\begin{array}{c} \frac{\partial E}{\partial y_{i}^{1-1}}=\sum w_{ij}^{1-1}\frac{\partial E}{\partial x_{j}^{1}}, \end{array}$$

where *w*_*ij*_^1−1^ is weight connected to input *x*_*j*_^1^ in next layer. Then, until input to the first completely linked layer is reached, (7) and (8) are repeated, resulting in the network's higher reasoning [36], or dense layers, training on one training sample. (9) represents the change in weight, which is supplementary to old weight:

(24) $$\begin{array}{c} \Delta w_{ij}^{1-1}=-\eta \frac{\partial E}{\partial y_{i}^{|-1}}, \end{array}$$

where *η* is the learning rate.

#### 3.1.7. Backpropagation-Max Pooling Layers

Backpropagation in convolutional layers is varied from that in the FC layer. Gradients for each weight in FC layers must be modified for the current layer. Since convolutional layer shares weights, each *x*_*i*,*j*_^−1^ expression with weight *w*_*ab*_ must be included. The gradient component for individual [37] weights are computed using the chain rule in the following way: *∂E*/*∂w*_*ab*_. This entails calculating affection of the loss function *E* based on a single pixel change in the weight kernel:

(25) $$\begin{array}{c} \frac{\partial E}{\partial w_{ab}}=\sum_{i=0}^{N-m}\sum_{j=0}^{N-m}\frac{\partial E}{\partial x_{ij}^{1}}\frac{\partial x_{ij}^{1}}{\partial w_{ab}}, \end{array}$$

where *∂x*_*ij*_^1^/*∂w*_*ab*_=*y*_(*i*+*a*)(*j*+*b*)_^1−1^

This is evaluated by utilizing chain rule again as in the following:

(26) $$\begin{array}{c} \frac{\partial E}{\partial x_{ij}^{1}}=\frac{\partial E}{\partial y_{ij}^{1}}\frac{\partial y_{ij}^{1}}{\partial x_{ij}^{1}}=\frac{\partial E}{\partial y_{ij}^{1}}\frac{\partial }{\partial x_{ij}^{1}}\left(\sigma \left(x_{ij}^{1}\right)\right)=\frac{\partial E}{\partial y_{ij}^{1}}\sigma^{\prime }\left(x_{ij}^{1}\right). \end{array}$$

Since the error at the current layer is already known, deltas may be simply determined by calculating the derivative of activation function. The activation function is max(0; *x*_*ij*_^1^) answer one or zero except for *x*_*ij*_^1^=0 when its derivative is not defined [38]. Following that, error must be transmitted to the preceding tier. This is accomplished once more by utilizing chain rule as shown in the following equation:

(27) $$\begin{array}{c} \sum_{a=0}^{m-1}\sum_{b=0}^{m-1}\frac{\partial E}{\partial x_{\left(1-a\right)\left(j-b\right)}^{1}}\frac{\partial x_{\left(1-a\right)\left(j-b\right)}^{1}}{\partial y_{jj}^{-1}}=\sum_{a=0}^{m-1}\sum_{b=0}^{m-1}\frac{\partial E}{\partial x_{\left(1-a\right)\left(j-b\right)}^{1}}w_{ab}. \end{array}$$

This equation represents a convolution in which *w*_*ab*_ has been flipped along both axes. It is also worth noting that this will not work for values at the top as well as the bottom.

#### 3.1.8. SVC (Support Vector Classifier)

Consider set *x*={*xi*1, *x*2,…, *xn*}with *xi* ∈ *ℜp* has a convincing pattern, that is grouped into positive class and negative class. The data are then considered as follows:

(28) $$\begin{array}{c} w.xi+b=0, \end{array}$$

where *w* is weights vector and *b* is scalar.

The problem of hyperplane *H*0 is same as finding optimal split field with the biggest margin value, which is expressed as follows:

(29) $$\begin{array}{c} \min\;1\;2\;\left\|w\right\|\;2\\ yi\left(wT.xi+\right)\geq 1,i=1,\ldots ,n. \end{array}$$

The linear case data in (29)classification nicely demonstrates how data can be divided into two types. Therefore, the slack variable *si* needs to be added so that *yi*(*wT*.*xi*+) ≥ 1 − *si* is obtained.

Following functions (29) can be used to solve the problem in equation as follows:

(30) $$\begin{array}{c} \min\;1\;2\;\left\|w\right\|2+C\left(\sum \sin\;i=1\right), \end{array}$$

with constrains

(31) $$\begin{array}{c} yi\left(wT.xi+\right)\geq 1-si,i=1,\ldots ,n.\;and\;si\geq 0\text{ for }\forall . \end{array}$$

C helps to reduce the model's complexity and minimize training errors. The optimization issue in equations (11)–(13) is written as an optimization [39] issue without constraints in (32) using the Lagrange function, as follows:

(32) $$\begin{array}{c} \min Lp\left(w,b,s,a\right)=1\;2\;\left\|w\right\|\;2+C\left(\sum \sin\;i=1\right)+\sum \alpha i\left(1-\left(yi\left(wT.xi+\right)-si\right)\right)ni=1. \end{array}$$

Non-negative variables are known as Lagrange Multiplier where ≥ 0. Goal of (14) is to reduce *Lp* to *w* and *b* while simultaneously increasing *Lp* to *w*. The dual issue of (14) can be solved using partial derivatives *Lp* to *w*, b, and *s* as follows:

(33) $$\begin{array}{c} \text{maks }L_{d}=\sum_{i=1}^{n}a_{i}-\frac{1}{2}\sum_{i=1}^{n}\sum_{i=1}^{n}a_{i}a_{j}y_{i}y_{j}\left(x_{i},x_{j}\right), \end{array}$$

with constraints

(34) $$\begin{array}{c} 0\leq a_{i}\leq C,\text{with }i=1\text{,}\ldots \text{,}n\\ \text{and}\sum_{i=1}^{n}a_{i}y_{i}=0. \end{array}$$

#### 3.1.9. Gaussian NB (Naives Bayes)

Nave Bayes is a simple and quick classification method that relies on the Bayes theorem and is expressed by the following:

(35) $$\begin{array}{c} P\left(Y\right)=\frac{P\left(X\right)P\left(X\right)}{P\left(Y\right)}. \end{array}$$

This classifier assumes that each variable contributes equally to the outcome on its own. Every characteristic is now independent of the others, and output is likewise affected by the same weight. As a result, the Nave Bayes theorem cannot be applied to real-world problems, and when this approach is utilized, only poor accuracy is obtained. As a result, Gaussian NB is utilized, which assumes that features have a normal distribution. Features have a conditional probability and are presumed to be Gaussian. Equation (36) gives the Gaussian NB as follows:

(36) $$\begin{array}{c} P\left(y\right)=\frac{1}{\sqrt{2\pi \sigma 2y}}\text{exp exp}\left(\frac{-{\left(xi-\mu y\right)}^{2}}{2\sigma^{2}}\right). \end{array}$$

## 4. Performance Analysis

This section compares the suggested strategy for ovarian cancer diagnosis to existing methods and analyses the performance analysis. The model's performance is represented by a confusion matrix that includes true negatives, true positives, false negatives, and false positives.

### 4.1. Database Description

The suggested classifier was tested on single-cell blood smear samples obtained from the Cancer Imaging Archive database [40]. Cropped sections of epithelial cells, germ cells, and stromal cells can be found in Cancer Imaging Archive database. The Cancer Imaging Archive database's grey level attributes are virtually identical to Cancer Imaging Archive database, but with a larger dimension.

The confusion matrix of Gaussian NB employing FaRe-ConvNN is shown in Figure 5 above, where rows indicate predicted class and columns represent an actual class of ovarian cancer data. Trained network that is correctly and erroneously classified is represented by the diagonal blue and white cells. The right-hand column represents each anticipated class, whereas the bottom row reflects each actual class' performance [41]. This confusion matrix plot for Gaussian NB utilizing FaRe-ConvNN reveals that the overall classification performance is 98.69 percent correct.

The confusion matrix of SVC employing FaRe-ConvNN is shown in Figure 6, with rows and columns indicating predicted as well as actual classes. This SVC confusion matrix plot utilizing FaRe-ConvNN reveals that total classification accuracy is 97.39 percent. The anticipated class is represented by the right-hand column, while the performance of each actual class is represented by the bottom row. To make it easier to examine the performance, zeroes are added here [42]. Few couples are frequently misidentified as a result of this confusion matrix. The analysis of SVC, as well as Gaussian NB with various specifications, is shown in Table 2.

Graphical depiction based on settings for Gaussian NB as well as SVM utilizing FaRe-ConvNN is shown in Figure 7. Precision, recall/sensitivity, and specificity are the metrics that have been determined in percent. SVC precision is 95.96 percent, whereas Gaussian NB precision is 97.7 percent, with FR-CNN enhancing precision in Gaussian NB. For recall/sensitivity, SVC is 94.31 percent and Gaussian NB is 97.7 percent, while for specificity, SVC is 97.39 percent and Gaussian NB is 98.69 percent using FaRe-ConvNN. The Gaussian NB technique in classification utilizing FaRe-ConvNN delivers an improved predicted class in ovarian cancer detection, as discussed above. The parametric values acquired by various approaches are compared in Table 3.

Figure 8 compares existing and proposed techniques in terms of precision, recall, and specificity. CNN [43] has an accuracy of 81.91 percent, DCNN has an accuracy of 89.19 percent, KNN has an accuracy of 78.45 percent, SVC has an accuracy of 95.96 percent, and Gaussian NB has an accuracy of 97.7 percent. CNN has a recall of 79.02 percent, DCNN has a recall of 88.28 percent, KNN has a recall of 74.19 percent, SVS has a recall of 94.31 percent, and Gaussian NB has a recall of 97.7 percent. CNN has 82.93 percent specificity, DCNN has 91.91 percent, KNN has 75.33 percent, SVC has 97.39 percent, and Gaussian NB has 98.69 percent. SVC and Gaussian NB with FR-CNN have outperformed all other approaches suggested.

## 5. Conclusion

In comparison to existing methodologies, the classification method of both SVC, as well as Gaussian NB utilizing FaRe-ConvNN, delivers a precision value of more than 95%, according to the performance analysis. Utilizing this proposed FaRe-ConvNN, 97 percent to almost 99 percent precision was acquired from the projected class utilizing this classification technique. Based on the results of the suggested method, it can be stated that this OC detection classification method is a significant contribution to the medical sector, assisting clinicians in making more precise decisions and treating patients more effectively. There is still scope for research contribution that too in the experimentation of different deep learning models and their hyperparameters optimization for achieving promising and trustable results. Also, intermediate results of CNN can be analyzed and further inferences can be derived for further research.

## Figures and Tables

**Figure 1:** Normal ovary and types of ovarian cancer.

**Figure 2:** Proposed methodology for the classification of ovarian cancer.

**Figure 3:** Example of max-pooling.

**Figure 4:** FR-CNN network with RPN.

**Figure 5:** Confusion matrix of Gaussian NB using FaRe-ConvNN.

**Figure 6:** Confusion matrix of SVC using FaRe-ConvNN.

**Figure 7:** Comparison of various parameters.

**Figure 8:** Comparison of various algorithms.

**Algorithm 1:** ROI segmentation with FaRe-ConvNN for Classification.

**Table 1:** Comparative analysis for proposed and existing techniques.

Study references	Techniques	Binary or multiclass	Modules	Accuracy	Other parameters
[9]	IABC-EMBOT, IHM-FFNN, PSO-RM, ABCO-BCD AND DNN-BCD	Binary	Negative, positive	0.975	—
[10]	FNN, ANFIS, ANNFIS	Binary	Negative, positive	0.92	Precision 0.944, recall 0.944
[11]	Deep type, state of the art	Multiclass	Normal, luminal A, B, basal and HER2	—	—
[12]	BPNN	Binary	Mutant as well as non-mutant sequences	0.998	Sensitivity = 0 Specificity = 0
[13]	CNN	Multiclass	—	0.956	—
[14]	DA	Multiclass	—	0.95	—
[15]	DNN + attention method	Multiclass	—	0.87	—
[16]	GCN	Multiclass	—	0.919	AUC = 0.84
[17]	DNN + SVM	Multiclass	Binary, miotic/non	0.83	F-score = 0.556 Accuracy = 0.8319
[18]	DNN	Multiclass	4 classes	0.97 by SVM	AUC = 0.82, accuracy = 0.8682
[19]	DL + ML	Multiclass	Auxiliary lymph node status, binary, cancer or not	0.84	Accuracy:0.98, AUC = 0.93
[21]	DL + ML	Multiclass	Binary, cancer or not	0.84	AUC:0.84

**Table 2:** Comparison of SVC and Gaussian NB classifiers.

Parameters	SVC (%)	Gaussian NB (%)
Precision	96.97	96.7
Specificity	98.40	97.68
Recall/Sensitivity	95.32	96.7

**Table 3:** Comparative Analysis of various techniques.

Parameters	KNN (%)	CNN (%)	DCNN (%)	SVC (%)	Gaussian NB (%)
Precision	90.12	80.90	90.10	96.11	97.7
Recall/Sensitivity	75.20	80.25	89.21	95.26	97.7
Specificity	96.30	85.13	90.10	96.32	98.69

## Data Availability

The data that support the findings of this study are available on request from the corresponding author.

## References

[1] Landrum L. M., Java J., Mathews C. A. (2013). Prognostic factors for stage III epithelial ovarian cancer treated within traperitoneal chemotherapy: a Gynecologic Oncology Group study. *Gynecologic Oncology*.

[2] Mangone L., Mandato V. D., Gandolfi R., Tromellini C., Abrate M. (2014). The impact of epithelial ovarian cancer diagnosis on women’s life: a qualitative study. *European Journal of Gynaecological Oncology*.

[3] Bhp (2017). Health survey by the bureau of health promotion (BHP). https://cris.hpa.gov.tw/pagepub/Home.aspx.

[4] Shafi U., Sharma S. (2019). Ovarian cancer detection in MRI images using feature space and classification method. *International Journal of Recent Technology and Engineering*.

[5] Bhardwaj H., Tomar P., Sakalle A., Bhardwaj A. Classification of extraversion and introversion personality trait using electroencephalogram signals.

[6] Alnuaim A. A., Zakariah M., Alhadlaq A. (2022). Human-computer interaction with detection of speaker emotions using convolution neural networks. *Computational Intelligence and Neuroscience*.

[7] Malik H., Fatema N., Alzubi J. A. (2021). *AI and Machine Learning Paradigms for Health Monitoring System: Intelligent Data Analytics*.

[8] Nolen B. M., Lokshin A. E. (2011). Screening for ovarian cancer: old tools, new lessons. *Cancer Biomarkers*.

[9] Liang C., Peng L. (2013). An automated diagnosis system of liver disease using artificial immune and genetic algorithms. *Journal of Medical Systems*.

[10] Bhardwaj H., Tomar P., Sakalle A., Acharya D., Badal T., Bhardwaj A. (2022). A DeepLSTM model for personality traits classification using EEG signals. *IETE Journal of Research*.

[11] Alnuaim A. A., Zakariah M., Shukla P. K. (2022). Human-computer interaction for recognizing speech emotions using multilayer perceptron classifier. *Journal of Healthcare Engineering*.

[12] Alzubi J. A. (2020). AI and Machine Learning Paradigms for Health Monitoring System. *Intelligent Data Analytics, 1E. Studies in Big Data*.

[13] Jelovac D., Armstrong D. K. (2011). Recent progress in the diagnosis and treatment of ovarian cancer. *CA: A Cancer Journal for Clinicians*.

[14] Sakalle A., Tomar P., Bhardwaj H., Acharya D., Bhardwaj A. (2021). An analysis of machine learning algorithm for the classification of emotion recognition. *Soft Computing for Problem Solving*.

[15] Karbalay-Doust S., Noorafshan A. (2012). Stereological estimation of ovarian oocyte volume, surface area and number: application on mice treated with nandrolone decanoate. *Folia Histochemica et Cytobiologica*.

[16] Alnuaim A. A., Zakariah M., Shashidhar C. Speaker gender recognition based on deep neural networks and ResNet50. *Wireless Communications and Mobile Computing*.

[17] İnik Ö, Ceyhan A., Balcioglu E., Ulker E. (2019). A new method for automatic counting of ovarian follicles on whole slide histological images based on convolutional neural network. *Computers in Biology and Medicine*.

[18] Mazzini M., Giorgi F. (1985). The follicle cell-oocyte interaction in ovarian follicles of the stick insect Bacillus rossius (Rossi): (Insecta: phasmatodea). *Journal of Morphology*.

[19] González-Reyes A., St Johnston D. (1998). Patterning of the follicle cell epithelium along the anterior-posterior axis during Drosophila oogenesis. *Development (Cambridge, United Kingdom)*.

[20] Kose U., Deperlioglu O., Alzubi J., Patrut B. (2021). *Deep Learning for Medical Decision Support Systems*.

[21] Sridhar C., Pareek P. K., Kalidoss R., Jamal S. S., Shukla P. K., Nuagah S. J (2022). Optimal medical image size reduction model creation using recurrent neural network and GenPSOWVQ. *Journal of Healthcare Engineering*.

[22] Drosophila Oogenesis (2018). *The Welcome/CRC Institute and Department of Genetics*.

[23] Browne C. L., Werner W. (1984). Intercellular junctions between the follicle cells and oocytes ofXenopus laevis. *Journal of Experimental Zoology*.

[24] Pareek P. K., Sridhar C., Kalidoss R. (2022). IntOPMICM: intelligent medical image size reduction model. *Journal of Healthcare Engineering*.

[25] Wu M., Yan C., Liu H., Liu Q. (2018). Automatic classification of ovarian cancer types from cytological images using deep convolutional neural networks. *Bioscience Reports*.

[26] Rayan R. A., Zafar I., Tsagkaris C. Deep learning for health and medicine. *Deep Learning for Personalized Healthcare Services*.

[27] Vasavi G., Jyothi S. Classification and detection of ovarian cysts in ultrasound images.

[28] Shukla P. K., Zakariah M., Hatamleh W. A., Tarazi H., Tiwari B. (2022). AI-DRIVEN novel approach for liver cancer screening and prediction using cascaded fully convolutional neural network. *Journal of Healthcare Engineering*.

[29] Schorge J. O., Modesitt S. C., Coleman R. L. (2010). SGO White Paper on ovarian cancer: etiology, screening and surveillance. *Gynecologic Oncology*.

[30] Hiremath P. S., Tegnoor J. R. (2013). Automated ovarian classification in digital ultrasound images. *International Journal of Biomedical Engineering and Technology*.

[31] Nawgaje D. D., Kanphade R. D. (2012). Hardware implementation of genetic algorithm for ovarian cancer image segmentation. *Proceedings of the International Journal of Soft Computing and Engineering (IJSCE)*.

[32] Kavitha S. (2021). Dr vidyaathulasiraman, “identification of proper machine learning classification model based on image annotation technique. *Annals of R.S.C.B*.

[33] Khan B., Shukla P. K., Ahirwar M. K., Mishra M., Rani G., Tiwari P. (2021). Strategic analysis in prediction of liver disease using different classification algorithms. *Handbook of Research on Disease Prediction through Data Analytics and Machine Learning*.

[34] Schwartz D., Sawyer T. W., Thurston N., Barton J., Ditzler G. (2022). Ovarian cancer detection using optical coherence tomography and convolutional neural networks. *Neural Computing & Applications*.

[35] Kowalski P. A., Błoniarz J., Chmura Ł., Cornejo M. E., Kóczy L. T., Medina-Moreno J., Moreno-García J. (2022). Convolutional neural networks in the ovarian cancer detection. *Computational Intelligence and Mathematics for Tackling Complex Problems 2 Studies in Computational Intelligence*.

[36] Krishnamoorthi R., Joshi S., Almarzouki H. Z. (2022). A novel diabetes healthcare disease prediction framework using machine learning techniques. *Journal of Healthcare Engineering*.

[37] Saba T. (2020). Recent advancement in cancer detection using machine learning: systematic survey of decades, comparisons and challenges. *Journal of Infection and Public Health*.

[38] Ali S., Li J., Pei Y., Khurram R., Rehman K. u., Rasool A. B. (2021). State-of-the-Art challenges and perspectives in multi-organ cancer diagnosis via deep learning-based methods. *Cancers*.

[39] Mikdadi D., O’Connell K. A., Meacham P. J. (2022). Applications of artificial intelligence (AI) in ovarian cancer, pancreatic cancer, and image biomarker discovery. *Cancer Biomark*.

[40] Mahmood T., Li J., Pei Y., Akhtar F., Imran A., Rehman K. U. (2020). A brief survey on breast cancer diagnostic with deep learning schemes using multi-image modalities. *IEEE Access*.

[41] Zebari A., Ahmed Ibrahim D., Qader Zeebaree D. (2021). Systematic review of computing approaches for breast cancer detection based computer aided diagnosis using mammogram images. *Applied Artificial Intelligence*.

[42] Motwani A., Shukla P. K., Pawar M., Reddy V. S., Prasad V. K., Wang J., Reddy K. T. V. (2021). Novel machine learning model with wrapper-based dimensionality reduction for predicting chronic kidney disease risk. *Soft Computing and Signal Processing Advances in Intelligent Systems and Computing*.

[43] NCI Welcome to The Cancer Imaging Archive. https://www.cancerimagingarchive.net/.

